RETRACTED

# Expression and Clinical Significance of Ki67 and SOX2 in Colorectal Cancer

**DOI:** 10.1155/2023/3783631

**Published:** 2023-07-07

**Authors:** Bo Hu, Xinfu Song, Weiji Ding, Hailong Wang, Huali Cai, Zhengjie Huang

**Affiliations:** ^1^Department of Gastrointestinal Surgery, Xiamen Humanity Hospital Fujian Medical University, Xiamen 361000, China; ^2^The Third Clinical Medical College, Fujian Medical University, Fuzhou 350122, China

## Abstract

The purpose of the paper is to explore the expression levels and clinical significance of Ki67 and sex-determining region Y-box 2 (SOX2) in colorectal cancer. From January 2013 to December 2016, 176 patients with colorectal cancer who were pathologically diagnosed after surgery in the Department of General Surgery in Xiamen Chinese Medical Hospital are included in this study. The pathological parameters, including gender, age, pathological stage, depth of tumor invasion, lymph node metastasis, and distant metastasis, are recorded. Immunohistochemistry is used to detect the correlation between Ki67 and Sox2 protein expression and clinicopathological parameters in colorectal cancer. Immunohistochemistry shows that in each stage of colorectal cancer, the positive rate of SOX2 is higher than that of Ki67, and the sensitivity of SOX2 is relatively high. Moreover, the levels of Ki67 and SOX2 in the cancerous tissues are not related to gender, age, lymph node metastasis and distant metastasis (*p* > 0.05).

## 1. Introduction

Colorectal cancer is one of the most common malignant tumors in the digestive system. Its incidence has an increasing tendency year by year, and its morbidity and mortality are ranked third and fourth worldwide, respectively [1, 2]. In China, with the change of modern lifestyle, the age of onset is becoming younger and younger [3]. Both environmental factors and genetic factors affect the occurrence and development of colorectal cancer, which is closely related to abnormal cell proliferation and apoptosis [4]. In recent years, with the rapid advancement of medical molecular biotechnology, research studies on various tumor-related factors have continued to deepen. However, there is still a lack of specific molecular markers that can effectively monitor the occurrence, development, and prognosis of colorectal cancer.

Ki67, a cellular proliferation marker, is mainly located in the nucleus. Because of its short half-life and because it is not easily affected by various growth factors, many researchers have taken Ki67 as an auxiliary indicator to monitor the proliferation activity of tumor cells in various systems [5]. However, in the studies of colorectal cancer related clinical data, the scholars have different points on Ki67. Nadya et al. have shown that Ki67 is associated with the pathological type and tumor differentiation of colorectal cancer, but not to the patient's gender, age, tumor volume, infiltration degree, tumor stage, lymph node metastasis, and vascular invasion [6]. Sex determining region Y (SRY)-box 2 (SOX2) is a member of the SOX family. In recent years, SOX2 has been found to be overexpressed in the tumor tissues of breast cancer, pancreatic cancer, and gastric cancer [7, 8]. Ardeshir et al. have suggested that SOX2 may be related to the age of onset, race, tumor morphology, stage, and lymph node metastasis of colorectal malignant tumors [9]. Nevertheless, its specific role and mechanism in colorectal cancer have not been fully understood.

RETRACTED

Therefore, the purpose of this study is to explore the correlation between the expressions of Ki67 and SOX2 and the clinicopathological features of patients with colorectal cancer so as to provide a corresponding theoretical basis for the clinical diagnosis, treatment, and prognosis of colorectal cancer.

The remainder of this paper is organized as follows: Section 2 presents the subjects and methods.  Section 3 describes western blotting and immunohistochemistry. Statistical analysis results are explained in Section 4.  Section 5 provides the clinical result analysis. Finally, the conclusions of this study and some future recommendations are given in Section 6.

## 2. Subjects and Methods

This paper has been approved by the Ethics Committee of Xiamen Chinese Medical Hospital. All patients signed informed consent. From January 2013 to December 2016, 176 patients with colorectal cancer who were pathologically diagnosed after surgery in the Department of General Surgery in Xiamen Chinese Medical Hospital are included in this study. The staging of colorectal cancer is based on the newly revised TNM staging standard of colorectal cancer by the American Joint Committee on Cancer (AJCC) in 2010. All patients underwent surgical resection of the tumor. All tumor tissue samples are confirmed by postoperative histopathology. Patients with colorectal cancer are divided into the early stage (I) group (*n* = 29) and the middle-advanced stage (II + III + IV) group (*n* = 147). The distant cancer tissue is defined as the control group.

The pathological parameters, including gender, age, pathological stage, depth of tumor invasion, lymph node metastasis, and distant metastasis, are recorded. The surgically resected malignant tumor specimens are removed from the body within 30 min after being isolated from the body. The distant cancer tissues, 5 cm away from the tumor edge (control tissues), are taken under aseptic conditions. Then, the cancerous tissues without necrosis are cut from the tumor tissues. The tissue samples are put into a 1.5 mL EP tube without RNA and DNase and then transferred to −80°C refrigerator for storage.  Table 1 shows the primer sequences provided by Sangen Biotechnology Co., Ltd.

RETRACTED

## 3. Western Blotting and Immunohistochemistry

A total of 8 g of tissues are homogenized in 500 *μ*l of cold RIPA buffer (Beyotime Institute of Biotechnology, Shanghai, China). The total protein is centrifuged at 15,000 × g for 15 min at 4°C. Supernatants are collected, and protein concentration is measured using a modified BCA protein concentration assay kit (Beijing Kangwei Century Biotechnology Co., Ltd., Beijing, China) in accordance with the manufacturer's protocol. An equal amount of protein (20 *μ*g) is separated by SDS-PAGE (BIO-RAD Co., California, USA) and transferred to a nitrocellulose membrane (Pall Co., NY, USA). The membrane is blocked for 1 h at room temperature with nonfat dried milk or bovine serum albumin (BSA) (Sangon Biotech Inc., Shanghai, China). The membrane is incubated with the primary antibodies (anti-Ki67 antibody (BOSTER Biological Technology Co., Ltd., Wuhan, China), anti-SOX2 antibody (Abcam Technology, Cambridge, UK), and anti-*β*-actin antibody (ZSGB Biotech Co., Ltd., Beijing, China)) overnight at 4°C. The membrane is then incubated with the second antibody (Beyotime Institute of Biotechnology, Shanghai, China) for 1h at room temperature and exposed to ECL Western Blotting Substrate reagent (Tsea Biotech Co., Shanghai, China). Molecular Imager Chemi Doc XRS (BIO-RAD Co., California, USA) and JS-780 automatic gel imaging analysis systems are used for blotting and quantitative analysis. *β*-actin is used as the internal control.

All immunohistochemical specimens are fixed in 10% formalin solution (Xilong Chemical Co., Ltd., Shantou, China) for 24 h, embedded in a paraffin embedding machine, and cut into 4 *μ*M sections. The sections are stained by immunohistochemistry with a commercial kit (Fuzhou Maixin Biotechnology Development Co., Ltd., Fuzhou, China). The main experimental steps are as follows: after paraffin sections are dewaxed and hydrated, the antigen is repaired by high-pressure heating with sodium citrate solution for 2 min, cooled naturally at room temperature. Each section is treated with a 3% H_2_O_2_ solution for 10 min to block the activity of endogenous peroxidase. Each section is dripped with nonimmune rat serum (Shanghai Yuanmu Biotechnology Co., Ltd., Shanghai, China) to reduce nonspecific staining. The first antibodies (anti-Ki67 antibody (BOSTER Biological Technology Co. Ltd., Wuhan, China), anti-SOX2 antibody (Abcam Technology, Cambridge, UK), and anti-*β*-actin antibody (ZSGB Biotech Co., Ltd., Beijing, China)) are added and incubated overnight at 4°C. After PBS cleaning, they are added with biotin labeled secondary antibody (ZSGB Biotech Co., Ltd., Beijing, China) and incubated at 37°C for 30 min. DAB is added for color development, and then hematoxylin staining solution is used to redye the sections. The sections are sealed with conventional dehydrated neutral resin, and the dyeing state is observed under the optical microscope (OLYMPUS BX41, OLYMPUS, Tokyo, Japan).

RETRACTED

The scoring methods of antigen staining expression included comprehensive staining intensity and the number of stained cells. The grading standard of staining intensity is as follows: Grade 0, no staining; Grade 1, weak staining; Grade 2, medium staining; and Grade 3, strong staining. The number of stained cells is scored according to the proportion of positive cells in each section. The proportion of positive cells is the average number of counts in each visual field (four visual fields). In Grade 0, the number of positive cells is 0%; in Grade L, the number of positive cells is less than 25%; in Grade 2, the number of positive cells is 25%–50%; in Grade 3, the number of positive cells is 50%–75%; and in Grade 4, the number of positive cells is more than 75%. Histological score = intensity score of staining × percentage score of positive cells. The total score is 12 points. (−) is 0 point, (+) is 1–4 points, (++) is 5–8 points, and (+++) is 9–12 points. (+), (++), and (+++) are defined as positive expression.

All experiments are repeated three times with the same sample. Statistical analysis is made by software SPSS26.0 (International Business Machines, corp., Armonk, NY, USA). All the data are expressed as the means ± standard deviation (SD). The correlation between qPCR data is analyzed by the Pearson correlation. The immunohistochemical expression and clinicopathological data are analyzed by the *χ*^2^ test. Differences are considered statistically significant when *p* < 0.05.

## 4. The Clinical Experimental Results

### 4.1. The mRNA Expression Levels of Ki67 and SOX2 in Control Tissues and Cancerous Tissues

The mRNA expressions of Ki67 and SOX2 in control tissues and cancerous tissues are detected by qPCR. Among 176 patients with colorectal cancer, Ki67 mRNA is highly expressed in the cancerous tissues of 120 patients (68.1%), while Ki67 mRNA expression in control tissues is downregulated or absent. In 109 patients with colorectal cancer, the SOX2 mRNA expression levels are significantly increased in cancerous tissues than in control tissues (*p* < 0.05).

Ki67 mRNA expression level in the cancerous tissues in patients with stage I are higher than that in patients with stage II, III, and IV ((9.14 ± 1.50) vs. (8.96 ± 1.61)). SOX2 mRNA expression levels in the cancerous tissues in patients with stage I are higher than those of patients with stage II, III, and IV ((9.96 ± 1.93) vs. (9.47 ± 1.76)). Moreover, there is a positive correlation between Ki67 and SOX2 in cancerous tissues, as shown in Figure 1. In cancerous tissue, the SOX2 mRNA level is significantly increased with the increased Ki67 mRNA level (*p* < 0.05), as shown in Table 2. Table 2 shows the correlation between the expression levels of Ki67 and Sox2 mRNA in cancer tissues. Figure 1 shows the correlation scatter of △ ct-ki67 and △ ct-sox2 data in cancer tissues of all patients.

RETRACTED

### 4.2. The Protein Expression Levels of Ki67 and SOX2 in Control Tissues and Cancerous Tissues

As shown in Figure 2, the Ki67 protein expression levels in the cancerous tissues are significantly increased than in the control tissues. Similarly, the SOX2 protein expression levels in the cancerous tissues are notably higher than in the control tissues. Figure 2 shows the protein expression levels of Ki67 and Sox2 in control and cancer tissues.

### 4.3. The Protein Expression Levels of Ki67 and SOX2 in Control Tissues and Cancerous Tissues Detected by Immunohistochemistry

As shown in Figure 3, Ki67 and SOX2 are both expressed in cancerous tissues. In colorectal cancer tissues of patients with stage I, the positive staining proportion of Ki67 is 37.9% (11/29) and that of SOX2 is 51.7% (15/29). In colorectal cancer tissues of patients with stage II, the positive staining proportion of Ki67 is 59.4% (41/69) and that of SOX2 is 72.5% (50/69). In the colorectal cancer tissues of patients with stage III, the positive staining proportion of Ki67 is 65% (39/60), and that of SOX2 is 70.0% (42/60). In colorectal cancer tissues of patients with stage IV, the positive staining proportion of Ki67 is 55.6% (10/18), and that of SOX2 is 77.8% (14/18), as shown in Table 3. The abovementioned results show that in each stage, the positive rate of SOX2 is higher than that of Ki67; that is, the sensitivity of SOX2 is relatively high. Table 3 shows the staining intensity of Ki67 and Sox2 in patients with colorectal cancer. Figure 3 shows the levels of Ki67 and Sox2 in control and cancer tissues detected by immunohistochemistry.

### 4.4. Correlation between Immunohistochemical Expression of Ki67 and Sox2 and Clinical Parameters

As shown in Table 4, the protein expression levels of Ki67 and SOX2 in the cancerous tissues are not related to gender, age, lymph node metastasis, and distant metastasis (*p* > 0.05). However, they are notably related to the TNM stage and the infiltration degree of colorectal cancer (*p* < 0.05). The higher the stage, the higher the positive rate of Ki67 and Sox2 protein expression (61.2%, *p* = 0.020 vs. 72.1%, *p* = 0.030). Table 4 shows the correlation between the immunohistochemical expression of Ki67 and Sox2 and clinical parameters.

RETRACTED

## 5. Data Analysis and Result Discussion

In recent years, with the rapid development of medical molecular biotechnology, scientists have made breakthroughs in the research of tumor-related factors. In this study, the expression levels of Ki67 and SOX2 in distant cancer tissues and cancerous tissues in patients with colorectal cancer are detected by qPCR, western blotting, and immunohistochemistry. We found that compared with distant cancer tissues, the mRNA and protein expression levels of Ki67 and SOX2 in distant cancer tissues are increased. Moreover, the SOX2 mRNA expression in cancerous tissues in each stage of colorectal cancer is positively correlated with the Ki67 mRNA expression, and the combined detection of the two has clinical significance in early prediction of the occurrence of colorectal cancer. Meanwhile, the protein levels of Ki67 and SOX2 are correlated with TNM staging and the depth of tumor invasion, suggesting that they may play an important role in the occurrence and development of colorectal cancer as potential cancer promoters.

Rahmanzadeh et al. believe that Ki67 is involved in the composition of rRNA required for ribosome in protein synthesis, so inhibiting the production of Ki67 protein can significantly affect the synthesis of cellular ribosomes. The high expression of Ki67 is closely related to the occurrence and development of malignant tumors, such as breast cancer, gastric cancer, lung cancer, cervical cancer, and urinary system malignancies. Lin et al. have found that the high expression of Ki67 is also closely related to the occurrence and development of colorectal cancer. However, in the study of the effect of Ki67 on colorectal cancer, different conclusions have been proposed by different scholars. Therefore, Ki67 is not suitable as a single indicator to judge the occurrence, development, and prognosis of colorectal cancer.

SOX2 is a transcription factor that encodes structurally related to sex determining region Y gene (SRY). At present, the main functions of SOX2 are as follows: (1) Participate in early embryonic development. Sox2, one of the key factors to maintain stem cell totipotency, plays an important role in maintaining stem cell self-renewal and multidirectional differentiation. If the cells begin to differentiate, SOX2 will stop expressing. According to this feature, it can be used as a molecular marker for pluripotent cell lineage. (2) Participate in the development of nerve tissues and organs. SOX2 exists in the early neural plate and neural tube, so it can be used as one of the signs of nervous system development. (3) Participate in the development of the human digestive tract. SOX2 can also affect the differentiation of gastric mucosal epithelial cells and regulate the expression of gastric differentiation markers. Its abnormal expression plays an important role in the process of gastric mucosal lesions and early gastric cancer. (4) Participate in the occurrence and development of tumors. More and more molecular biology studies suggest that the mutation and abnormal expression of the SOX2 gene are closely related to the occurrence and development of tumors in multiple systems (breast, pancreas, stomach, etc.). However, SOX2 has not achieved significant results in the occurrence, treatment, and prognosis of colorectal cancer until now.

RETRACTED

Lundberg et al. suggest that the expression of SOX2 and CDX2 in colorectal cancer tissues have a certain correlation, and the expression of SOX2 is regulated by the BRAF factor, which is related to the poor prognosis of patients with colorectal cancer. SOX2-positive tumor cells have strong metastasis. Jin et al. have found that the expression of miR-450b-5p is negatively correlated with the expression of SOX2. SOX2 could eliminate the inhibitory effect of miR-450b-5p on stem cells and chemical resistance of HT29 cells, representing the discovery of a new therapeutic target of colorectal cancer. Our results indicate that Ki67 and SOX2 are correlated in different stages of colorectal cancer. And the correlation in the early stages of colorectal cancer is greater than that in the middle and late stages of colorectal cancer. It is suggested that the increased mRNA expression of SOX2 and Ki67 may be an early event in the occurrence and development of colorectal cancer. The combined detection of SOX2 and Ki67 can jointly predict the development of colorectal cancer and may provide a theoretical basis for SOX2 as a detection indicator for screening early colorectal cancer. At the same time, SOX2 combined with Ki67 makes it possible to improve the early diagnosis rate of cancerization of adenoma tissues found in colonoscopy.

Moreover, we found that the protein expression levels of Ki67 and SOX2 are both expressed higher in cancerous tissues than in control tissues. It is the same as the results of Takahito et al., and they have found that in terms of tumor differentiation, ectopic gastrointestinal phenotype, neuroendocrine cell differentiation, and SOX2 expression are different in different colorectal laterally developing (transverse diffusion) tumors (LST).

RETRACTED

## 6. Conclusion

The immunohistochemical results showed that the positive rate of SOX2 is higher than that of Ki67 in each stage of colorectal cancer. Therefore, SOX2 is more sensitive than Ki67 in observing the occurrence and development of tumor and judging the prognosis. Meanwhile, the protein expression levels of Ki67 and SOX2 in the cancerous tissues are not related to gender, age, lymph node metastasis, and distant metastasis. However, they are notably related to the TNM stage and the infiltration degree of colorectal cancer. The results of combined qPCR and immunohistochemistry suggest that, consistent with the complex process of multigene, multistep, and multistage colorectal cancer, Ki67 and SOX2 may gradually progress to the increase of protein translation level from the abnormal overexpression of early transcription level. It suggests that their abnormal changes of posttranscription level may further aggravate with the occurrence and development of colorectal cancer. The combined detection of Ki67 and SOX2 can predict the development of colorectal cancer, especially as a detection indicator for screening early colorectal cancer.

## Figures and Tables

**Figure 1:** Correlation scatter of △ ct-ki67 and △ ct-sox2 data in cancer tissues of all patients.

**Figure 2:** The protein expression levels of Ki67 and Sox2 in control and cancer tissues.

**Figure 3:** The levels of Ki67 and Sox2 in control and cancer tissues detected by immunohistochemistry: (a) Ki67(−); (b) Ki67(+); (c) Ki67(++); (d) Ki67(+++); (e) SOX2 (−); (f) SOX2 (+); (g) SOX2 (++); (h) SOX2 (+++).

**Table 1:** The primer sequences provided by Sangen Biotechnology Co., Ltd.

Gene	Forward primer	Reverse primer
Ki-67	F5′-CTGACCCTGATGAGAGTGAGGGA-3′	R5′-ACTCTGTAGGGTCGAGCAGG-3′
SOX2	F5′-TGGACAGTTACGCGCACAT-3′	R5′-CGAGTAGGACATGCTGTAGGT-3′
*β*-actin	F5′-GAAGAGCTACGAGCTGCCTGA-3′	R5′-CAGACAGCACTGTGTTGGCG-3′

**Table 2:** The correlation between the expression levels of Ki67 and Sox2 mRNA in cancer tissues.

Items	Stages	Number	△Ct-SOX2	
			R	*P*
△Ct-Ki67	Stage I	29	0.444	<0.0001
	Stage II–IV	147	0.344	<0.0001

**Table 3:** The staining intensity of Ki67 and Sox2 in patients with colorectal cancer.

Items	Ki67				SOX2			
	−	+	++	+++	−	+	++	+++
Stage I	18	10	1	0	14	15	0	0
Stage II	28	32	9	0	19	45	5	0
Stage III	21	29	8	2	18	41	1	0
Stage IV	8	9	1	0	4	14	0	0

**Table 4:** The correlation between the immunohistochemical expression of Ki67 and Sox2 and clinical parameters.

Clinical parameters	Cases	Ki67			SOX2		
		Positive cases	*χ* ^2^	*p* values	Positive cases	*χ* ^2^	*p* values
Gender			0.104	0.747		0.042	0.839
Male	94	55			64		
Female	82	46			57		
Age			1.908	0.167		0.303	0.582
<60	95	50			67		
≥60	81	51			54		
TNM stage			5.374	0.020		4.685	0.030
I	29	11			15		
II + III + IV	147	90			106		
Infiltration degree			8.365	0.004		10.313	0.001
I + II	38	14			18		
III + IV	138	87			103		
Lymph node metastasis			0.114	0.739		0.761	0.383
Positive	18	11			14		
Negative	158	90			107		
Distant metastasis			3.103	0.078		1.340	0.247
Positive	104	54			68		
Negative	72	47			53		

RETRACTED

## Data Availability

The simulation experiment data used to support the findings of this study are available from the corresponding author upon request.
